The article "Upregulation of Actin-Related Protein 2 (ACTR2) Exacerbated the Malignancy of Diffuse Large B-Cell Lymphoma through Activating Wnt Signaling" was published in 2022. Journal: Comput Math Methods Med.

# Upregulation of Actin-Related Protein 2 (ACTR2) Exacerbated the Malignancy of Diffuse Large B-Cell Lymphoma through Activating Wnt Signaling

**DOI:** 10.1155/2022/9351921

**Published:** 2022-12-14

**Authors:** Dandan Chen, Lili Jiang

**Affiliations:** Department of Hematology, Nantong Haimen People's Hospital, China

## Abstract

This investigation mainly explores the roles of actin-related protein 2 (ACTR2) in diffuse large B-cell lymphoma (DLBCL). We first assessed the level of ACTR2 and its association with the overall survival (OS) of DLBCL. The results indicated that ACTR2 was upregulated in DLBCL and was associated with unfavorable prognosis of DLBCL. Next, the effect of ACTR2 knockdown or overexpression on DLBCL was evaluated *in vitro*. Our investigation revealed that ACTR2 depletion inhibited the malignant behaviors of DLBCL cells; whereas, ACTR2 abundance promoted those behaviors. Besides, ACTR2 activated the Wnt signaling in DLBCL and exerted its oncogenic influence on DLBCL through Wnt signaling *in vitro* and *in vivo*. To summarize, our study implicated that ACTR2 was a promising therapeutic target for DLBCL, which might become a novel direction to improve our understanding on DLBCL.

## 1. Introduction

Diffuse large B-cell lymphoma (DLBCL), the most common subtype of non-Hodgkin lymphoma (NHL) [1], is a type of lymphoid malignancy composed of highly proliferative large cells with basophilic cytoplasm, prominent nucleoli, and vesicular nuclei [2]. Based on the levels of genes related to the development of B cells, DLBCL can be divided into several subtypes, including germinal center B-cell (GCB) lymphoma, primary mediastinal B-cell lymphoma, and activated B-cell (ABC) lymphoma [3]. With the application of R-CHOP therapy as a standard treatment for DLBCL, great improvements have been made in the prognosis of DLBCL patients [4]. Nonetheless, the 5-year survival rate of DLBCL patients remains lower than 60% due to the refractory effect to initial treatment or relapses following routine therapies [5]. Therefore, it is still essential to deepen understanding on the biology and molecular mechanism of DLBCL to search for new therapeutic targets.

The actin-related protein 2/3 (ARP2/3) complex is the key nuclear in the branched actin cytoskeleton which participates in diverse cellular processes, including cell motility, vesicular trafficking, signaling, cytokinesis, and mechanical processes [6]. ACTR2 (also known as ARP2) is one of the two essential actin-associated proteins (ACTR2 and ACTR3) in the ARP2/3 complex [7]. In recent years, the dysregulation and functions of ACTR2 have been discovered in human diseases and cancers. For example, ACTR2/3 was downregulated in the serum-derived exosomes of patients diagnosed with Moyamoya disease [8]. ACTR2 was lowly expressed in essential thrombocytosis and has significant prognostic value [9]. ARPC2 was discovered to the abundantly expressed in hepatocellular carcinoma (HCC) and predicted unfavorable OS and progression-free survival of HCC [10]. Nevertheless, the prognostic significance and biological functions of ACTR2 in DLBCL have never been reported.

This study is aimed at stating the roles of ACTR2 in the progression of DLBCL by evaluating the expression, biological function, and underlying mechanism of ACTR2 in DLBCL. Our findings might provide novel insights in the understanding of DLBCL.

## 2. Materials and Methods

### 2.1. Cell Culture

DLBCL cell lines (U2932, SU-DHL-6, SU-DHL-8, and OCL-LY10) and human B lymphocyte (WIL2S) were bought from the Cell Bank of the Chinese Academy of Science (Shanghai). All cells were reserved in DMEM (HyClone), supplemented with 10% FBS (Gibco) and 1% penicillin–streptomycin solution at 37°C with 5% CO_2_.

### 2.2. Cell Transfection

shRNA against ACTR2 (shACTR2), the negative control (shNC), ACTR2 overexpression plasmid (pcDNA3.1/ACTR2), and empty pcDNA3.1 as control was purchased from GenePharma (Shanghai). DLBCL cells were transfected with vectors using Lipofectamine 2000 (Invitrogen) and subjected to drug selection in order to establish stable transfectants.

### 2.3. Western Blotting

Protein expressions were evaluated by western blot analysis. Briefly, equal amounts of proteins isolated from DLBCL cells or tissues were separated by 10% SDS-PAGE and transferred onto PVDF membranes which were first incubated with primary antibody against ARPC2, *β*-catenin, c-Myc, and cyclin D1 (Abcam) and then incubated with appropriate secondary antibodies for 1 h at room temperature. Protein bands were visualized with the ECL kit (Beyotime).

### 2.4. CCK-8 Assay

SU-DHL-8 and OCL-LY10 cells were seeded in the 96-well plates (1 × 10^4^ cells per well). 10 *μ*l CCK-8 solution was added to each well and incubated with the cells for 2 h. The optical density (OD) values were observed at a wavelength of 450 nm to assess proliferation of the treated cells.

### 2.5. Transwell

Transwell chambers (BD Biosciences) were used to assess migration and invasion of DLBCL cells. Cells in serum-free medium were seeded into the upper chambers (with Matrigel coating for cell invasion; no coating for cell migration). Medium containing 20% FBS was filled to the lower chambers as chemoattractant. 48 h after, the cells invaded/migrated through the membrane were fixed and stained in crystal violet. The stained cells were counted using a microscope (Olympus).

### 2.6. TUNEL

TUNEL assay was performed as previously described [11]. Briefly, the cell suspension was fixed in 4% paraformaldehyde for permeabilization. Then, the cells were incubated with the TUNEL mixture and counterstained with DAPI. Finally, the apoptotic cells were counted using a fluorescence microscope.

### 2.7. Xenograft Mouse Model

To develop OCL-LY10 xenograft, 4 weeks old BALB/c-nude mice (SLAC Laboratory Animal) were injected subcutaneously in the right abdomen with OCL-LY10 cells (1 × 10^7^) transfected with shNC or shACTR2. After 30 days, the mice were sacrificed and the weight of tumors were measured [12].

### 2.8. Statistical Analysis

Data are presented as the means ± SD. Each experiment was performed for no less than three times. Statistical comparisons were performed using Student's *t* test or one-way ANOVA between two groups or among more than two groups. The statistical significance level was set at *p* < 0.05. All statistics were performed by utilizing SPSS 18.0 (SPSS Inc.).

## 3. Results

### 3.1. ACTR2 Expression Was Elevated in DLBCL

A pancancerous analysis for the expression of ACTR2 in TCGA database indicated that ACTR2 was upregulated in 12 different types of cancers (BLCA, BRCA, CESC, CHOL, ESCA, HNSC, KIRC, LIHC, LUAD, LUSC, STAD, and UCEC) and downregulated in COAD and KICH (Figure 1(a)). Then ACTR2 expression was investigated in DLBCL; Figure 1(b) showed that ACTR2 was abundantly expressed in DLCBL tissues. Besides, Kaplan-Meier analysis implicated that high ACTR2 expression was associated with worse overall survival (Figure 1(c)). Moreover, western blot detected that level of ACTR2 was greatly elevated in DLBCL cells (U2932, SU-DHL-6, SU-DHL-8, and OCL-LY10) compared with that in WIL2S cells. In a word, ACTR2 was upregulated in DLBCL tissues and cells and correlated with unfavorable survival, implicating ACTR2 as a possible oncogene in DLBCL.

### 3.2. ACTR2 Silence Inhibited the Malignant Behaviors of DLBCL Cells

DLBCL cells (SU-DHL-8 and OCL-LY10) were selected for *in vitro* assays because those two cell lines exhibited particularly higher expressions of ACTR2. ACTR2 was silenced in SU-DHL-8 and OCL-LY10 cells and western blot showed markedly reduced level of ACTR2 (Figure 2(a)). After ACTR2 silencing, the proliferation of DLBCL cells was noticeably retarded (Figure 2(b)). Besides, the cells migrated and invaded to the lower transwell chamber were greatly reduced by depleting ACTR2 (Figures 2(c) and 2(d)). Moreover, the percent of apoptotic DLBCL cells increased remarkably following ACTR2 knockdown (Figure 2(e)). Taken together, the proliferation and metastasis of DLBCL cells were blocked by ACTR2 deficiency.

### 3.3. ACTR2 Overexpression Promoted the Malignancy of DLBCL Cells

To revalidate the role of ACTR2 in DLBCL, ACTR2 was overexpressed in SU-DHL-8 and OCL-LY10 cells (Figure 3(a)). The growth rate of SU-DHL-8 and OCL-LY10 cells was obviously augmented (Figure 3(b)). Moreover, the migration and invasion of DLBCL cells were greatly enhanced by ACTR2 overexpression (Figures 3(c) and 3(d)). In the meantime, ACTR2 abundance caused decreased apoptosis of SU-DHL-8 and OCL-LY10 cells (Figure 3(e)). To conclude, abundant ACTR2 expression promoted the progression of DLBCL *in vitro*.

### 3.4. ACTR2 Activates the Wnt Signaling in DLCBL

GSEA analysis identified the association between ACTR2 upregulation and the enrichment of Wnt signaling in DLBCL (Figure 4(a)). Wnt signaling has been widely reported to participate in the progression of human cancers, including DLBCL [13–16]. As shown in Figures 4(b) and 4(c), ACTR2 depletion and supplementation could decrease and increase the level of Wnt signaling-related proteins (*β*-catenin, c-Myc, and cyclin D1), respectively. Moreover, TCGA database showed remarkably elevated expression of *β*-catenin, c-Myc, and cyclin D1 in DLBCL tissues (Figures 4(d)–4(f)). Furthermore, a positive correlation between ACTR2 expression and the expression of CTNNB or c-Myc or CCND1 in DLBCL tissues was confirmed though using TCGA database (Figure 4(g)–4(i)). In sum, ACTR2 activated Wnt signaling in DLBCL.

### 3.5. Inhibition of Wnt Signaling Attenuates the Promotive Effect of ACTR2 on DLBCL Malignancy *In Vitro*

XAV939, an inhibitor of Wnt signaling, was introduced to perform rescue experiments. Firstly, ACTR2 overexpression greatly elevated the protein level of *β*-catenin, c-Myc, and cyclin D1 in DLBCL cells, but the introduction of XAV939 suppressed the elevation (Figure 5(a)). Results from functional assays demonstrated that the participation of XAV939 overturned the promotive impact of pcDNA3.1/ACTR2 transfection on the viability, migration, and invasion of DLBCL cells and the suppressive effect on DLBCL cell apoptosis (Figures 5(b)–5(f)). To summarize, ACTR2 accelerated the development of DLBCL *in vitro* through activating Wnt signaling.

### 3.6. ACTR2 Knockdown Blocked the Wnt Signaling to Suppress Tumor Growth

To validate the effects of ACTR2 *in vivo*, two groups of OCL-LY10 xenograft were constructed.  Figure 6(a) clearly showed that the volume and weight of tumors in shACTR2 group were noticeably lower than the control group. Besides, the levels of ACTR2 were obviously deficient in the tumors grown from ACTR2-silenced OCL-LY10 cells (Figure 6(b)). IHC assay further confirmed that the Ki-67 staining was greatly weakened in shACTR2 group of tumors (Figure 6(c)). Finally, western blot detected that the protein expression of *β*-catenin, c-Myc, and cyclin D1 was remarkably repressed by ACTR2 depletion (Figure 6(d)), implicating that ACTR2 deficiency could block the Wnt signaling *in vivo*. Collectively, silence of ACTR2 inhibited DLBCL tumor growth by blocking the Wnt signaling.

## 4. Discussion

Bioinformatics analysis has been widely employed to discover more effective biomarkers in improving the diagnosis and treatment of human diseases and cancers [17, 18], including DLBCL. For example, piRNA-30473 was uncovered to be upregulated in fresh DLBCL tissues using microarray analysis and proved to be a significant prognostic biomarker for DLBCL, and the knockdown of piRNA-30473 inhibited the tumorigenesis of DLBCL [19]. Higher CCND2 expression is associated with more efficient R-CHOP treatment and better prognosis of ABC-DLBCL [20]. High IQGAP2 level predicted shorter OS of DLBCL and was positively related to immunosuppressive gene expression in DLBCL [21]. The current investigation used TCGA database and uncovered the dysregulation of ACTR2 in 14 types of human cancer tissues in addition to DLBCL, suggesting its potential importance in cancer progression. We further evaluated its prognostic significance through Kaplan-Meier analysis which indicated that ACTR2 predicted worse OS in DLBCL. The oncogenic role of ACTR2 was also implicated by the greatly elevated protein levels in DLBCL cells.

In many cases, mRNAs exert the oncogenic effect through activating signaling pathways. For example, Liu et al. reported that SPAG5 upregulated survivin to accelerate the progression of gastric cancer through activation of the wnt/*β*-catenin pathway [22]. Cheng et al. revealed that FSTL1 has elevated expression in breast cancer and activated integrin *β*3/Wnt signaling to enhance the stemness and reduce chemosensitivity of breast cancer cells [23]. Xu et al. found that IGF2BP2 abundance in pancreatic cancer facilitated tumor growth by triggering the PI3K/Akt signaling [24]. Therefore, we hypothesized that ACTR2 could mediate the behaviors of DLBCL cells through certain signaling pathways. The relationship between ACTR2 and Wnt signaling was revealed through GSEA analysis. Wnt signaling pathway has been widely studied in human cancers and reported to play tumor-promotive roles in cancer progression, therefore considered as an effective therapeutic target [25, 26]. Noticeably, Wnt signaling has also been revealed to be involved in the development of DLBCL. For instance, GPNMB accelerated the malignancy of DLBCL by activating the YAP1-regulated Wnt/*β*-catenin signaling [27]. TIMD4 enhanced DLBCL cell viability via activating Wnt/*β*-catenin signaling [28]. MYC-induced lncRNA FIRRE upregulation exacerbated the malignancy of DLBCL through Wnt/*β*-catenin signaling [29]. Wnt pathways can be divided into *β*-catenin-dependent (canonical) and *β*-catenin-independent (noncanonical) Wnt signaling [30]. Previous reports indicated that canonical and noncanonical Wnt pathways might act differently in tumorigenesis, and they might also crosstalk in several cancers [31, 32]. Herein, the regulatory effect of ACTR2 on canonical Wnt signaling was investigated, and the results implicated that the upregulation of ACTR2 significantly augmented canonical Wnt signaling-related proteins in DLBCL cells. XAV939 is a tankyrase inhibitor that specifically targets the canonical Wnt pathway by increasing Axin protein expression, thereby stimulating *β*-catenin degradation [33]. Our results indicated that XAV939 reversed the effect of ACTR2 overexpression on the carcinogenesis of DLBCL, suggesting ACTR2 acted as an oncogene in DLBCL by triggering canonical Wnt pathway. Future studies on Wnt noncanonical pathway regulators and their interplay with the canonical pathway will be necessary to improve our knowledge on Wnt signaling in DLBCL.

Collectively, this study demonstrated that ACTR2 was abundant in DLBCL, which predicted worse OS. More importantly, the progression of DLBCL could be retarded through the knockdown of ACTR2 to block the Wnt signaling, implicating ACTR2 as a promising biomarker in the diagnosis and treatments of DLBCL.

## Figures and Tables

**Figure 1:** ACTR2 expression is significantly elevated in DLBCL and predicts worse OS. (a) Pancancer analysis of ACTR2 expression. (b) ACTR2 expression in DLBCL and normal tissues. (c) Kaplan-Meier analysis of the correlation between ACTR2 expression and OS in DLBCL. (d) Western blot detected ACTR2 expression in DLBCL cells.^∗^*p* < 0.05, ^∗∗^*p* < 0.01.

**Figure 2:** ACTR2 silencing blocks the malignant behaviors of DLBCL cells. ACTR2 was depleted in SU-DHL-8 and OCL-LY10 cells. (a) ACTR2 expression was evaluated by western blot assay. (b–e) The viability, migration, invasion, and apoptosis of DLBCL cells detected by CCK-8, transwell, and TUNEL assays.^∗∗^*p* < 0.01, ^∗∗∗^*p* < 0.001.

**Figure 3:** ACTR2 overexpression facilitates the malignant behaviors of DLBCL cells. ACTR2 was overexpressed in SU-DHL-8 and OCL-LY10. (a) ACTR2 expression was evaluated by western blot assay. (b–e) The viability, migration, invasion, and apoptosis of DLBCL cells detected by CCK-8, transwell, and TUNEL assays. ^∗∗^*p* < 0.01.

**Figure 4:** ACTR2 activates Wnt signaling in DLBCL. (a) GSEA enrichment analysis result. (b, c) Western blot detected the level of *β*-catenin, c-Myc, and cyclin D1 in SU-DHL-8 and OCL-LY10 cells after ACTR2 depletion or supplementation. (d–f) Levels of *β*-catenin (d), c-Myc (e), and cyclin D1 (f) between tumor and normal tissues in TCGA database. (g–i) The correlation between ACTR2 expression and the expression of *β*-catenin (g), c-Myc (h), and cyclin D1 (i) in DLBCL tissues.^∗∗^*p* < 0.01, ^∗∗∗^*p* < 0.001.

**Figure 5:** Wnt inhibitor overturns the promotive effect of ACTR2 abundance on DLBCL cellular activities. SU-DHL-8 and OCL-LY10 cells were transfected with pcDNA3.1, pcDNA3.1/ACTR2, or pcDNA3.1/ACTR2+XAV939. (a) Protein expression of *β*-catenin, c-Myc, and cyclin D1 was evaluated by western blot. (b–e) The viability, migration, invasion, and apoptosis of DLBCL cells detected by CCK-8, transwell, and TUNEL assays. ^∗^*p* < 0.05, ^∗∗^*p* < 0.01.

**Figure 6:** ACTR2 knockdown inhibits DLBCL tumor growth through blocking Wnt signaling. Xenograft tumors were developed from OCL-LY10 cells transfected with shNC or shACTR2. (a) Tumor volume and weight were observed. (b) Western blot detected the protein expression of ACTR2. (c) IHC detected the expression of Ki-67. (d) Western blot detected the protein expression of *β*-catenin, c-Myc, and cyclin D1.^∗∗^*p* < 0.01.

## Data Availability

No data were used to support this study.
